# Correlation between Transforming Growth Factor-*β* and Periapical Lesions in Patients with Chronic Apical Periodontitis

**DOI:** 10.1155/2022/2173434

**Published:** 2022-03-22

**Authors:** Xiujuan Li, Xuesong Han, Wenlei Yu, Xing Chen, Ying Wu, Linjie Lu

**Affiliations:** ^1^Department of Stomatology, Affiliated Hospital of Hangzhou Normal University, Hangzhou 310015, Zhejiang Province, China; ^2^School of Stomatology, Hangzhou Normal University, Hangzhou 311121, China

## Abstract

**Objective:**

To examine the expression of transforming growth factor-*β* (TGF-*β*) in the periapical granulation tissue and serum of patients with chronic apical periodontitis and to conduct immunohistochemical analysis so as to explore the relationship between TGF-*β* and the degree of periapical lesions.

**Methods:**

Periapical granulation tissues of 20 cases of chronic apical periodontitis were collected as the experimental group. Healthy gingival tissues without eruption of third molars of 5 cases were collected as the control group. Immunohistochemistry, enzyme-linked immunosorbent assay, and real-time PCR (RT-PCR) were utilized to determine the expression of TGF-*β* mRNA and protein, and the difference in the expression of TGF-*β* was compared between groups. In the experimental group, oral CBCT was taken to measure the periapical bone resorption area. Spearman's correlation method was applied to analyze the correlation between TGF-*β* protein and gene expression levels and periapical bone resorption area.

**Results:**

Immunohistochemistry and enzyme-linked immunosorbent assay demonstrated that the expression of TGF-*β* protein in chronic apical periodontitis tissue and serum was higher than that in the controls (*P* < 0.05). RT-PCR revealed that the expression of TGF-*β* mRNA was higher in chronic apical periodontitis tissue than that of the controls (*P* < 0.05). Spearman's correlation analysis showed that in the experimental group, the mRNA expression of TGF-*β* was positively correlated with the periapical bone resorption area (*P* < 0.01), and the protein expression level was not correlated with the periapical bone resorption area (*P* < 0.05).

**Conclusion:**

The increased expression of TGF-*β* in the periapical granulation tissue and serum of patients with chronic apical periodontitis has a certain correlation with the progression of periapical periodontitis. The correlation between TGF-*β* at the mRNA level and the degree of early stage disease as well as the high expression of TGF-*β* in inflammatory cells in immunohistochemistry have confirmed that TGF-*β* promotes bone resorption in early periapical periodontitis, and its mechanism of action deserves further investigation.

## 1. Introduction

Chronic apical periodontitis, a common and frequent oral disease in clinic, mainly occurs in the tissues around the tooth apex and is caused by infection, trauma, and other odontogenic factors [1]. At present, root canal therapy is the most commonly used and most effective therapy for treating chronic apical periodontitis. The prerequisite is to go through perfect root canal preparation and disinfection so as to prevent reinfection of the root canal and reduce the inflammatory response of the periapical tissue. The clinical symptoms of chronic apical periodontitis are not obvious, so chronic apical periodontitis is easy to be misdiagnosed and delayed. Under the stimulation of chronic inflammation and abscess, fibrous connective tissue around the tooth apex gradually presents apical periodontitis with fistula [2]. Chronic apical periodontitis is actually a kind of immune defense response, involving various inflammatory cells and cytokines. Therefore, we have performed a preliminary test to screen for various cytokines involved in periapical lesions. The results showed the increased expression of transforming growth factor-*β* (TGF-*β*) in the tissues of apical periodontitis. A previous study has demonstrated that the expression of TGF-*β* is correlated with periapical cysts treated within four years [3]. Some scholars have injected TGF-*β* into the joints of mice. It was found that numerous leukocytes and inflammatory factors infiltrated the articular cartilage in a short period and caused serious damage to the articular cartilage [4]. These studies provide theoretical supports to explore the expression of TGF-*β* in the granulation tissue of the sinus tract of chronic apical periodontitis patients. It is speculated that TGF-*β* exerts a crucial effect on the occurrence and development of chronic apical periodontitis, but its action mechanism needs to be further studied.

TGF-*β* has multiple roles in controlling cell proliferation and differentiation, wound healing, and immune system, plays a key role in pathology, such as the treatment of bone diseases, the induction of organ fibrosis and the regulation of the microenvironment of tumor cell growth, and promotes cancer cell apoptosis in the early stage of tumor [3–5]. A previous study has confirmed that TGF-*β* can induce the migration and differentiation of vascular endothelial cells and vascular smooth muscle. TGF-*β* has both vascular inhibitory and proangiogenic activities, and plays a dual role in angiogenesis [6]. The research on TGF-*β* in the field of oral cavity mainly focuses on controlling distraction osteogenesis through activating signaling pathways and promoting new bone formation, on TGF-*β* expression in salivary gland tumors, and on the reconstruction and remodeling of periodontal tissue during orthodontic tooth movement [7–9]. Few reports address the expression and role of TGF-*β* in human periapical periodontitis. Taken together, studying TGF-*β* expression in human chronic apical periodontitis tissue is of great significance for in-depth investigation of cytokines involved in the occurrence, development, and prognosis of chronic apical periodontitis.

This study observed and analyzed the expression of TGF-*β* in different degrees of chronic apical periodontitis from the levels of mRNA and protein, explored proinflammatory effect of TGF-*β* in chronic apical periodontitis, and provided new ideas for the development mechanism of chronic apical periodontitis.

## 2. Materials and Methods

### 2.1. Case Selection

Patients in the Department of Stomatology, Affiliated Hospital of Hangzhou Normal University, China, aged 18 to 65 years old, with a mean of (39.05 ± 13.00) years old, were recruited in this study. No statistical difference in the age was detected among all subjects. Inclusion criteria are as follows: (1) no vital organ dysfunction, no systemic diseases or pregnancy; (2) no antibiotics for at least 1 month; and (3) voluntarily signing informed consent. This experiment was approved by Ethics Committee of Affiliated Hospital of Hangzhou Normal University, China.

### 2.2. Group Assignment and Sample Collection

The granulation tissues of the sinus tract of 20 patients with chronic apical periodontitis were collected as experimental group. Inclusion criteria are as follows [10–12]: (1) X-ray films of the affected tooth revealed bone destruction in the apical region; (2) no response to pulp vitality test; (3) periodontal pocket depth <3 mm and not connected to the periapical and sub-bifurcation lesions; (4) can obtain the granulation tissue of the sinus tract connected to the tooth apex. Exclusion criteria are as follows: (1) other oral diseases or oral tumors; (2) combination of systemic disease or vital organ dysfunction; (3) a history of local or systemic medication (antibiotics and nonsteroidal anti-inflammatory drugs) within 1 month; (4) a history of root canal therapy or undergoing root canal therapy; and (5) periodontal ligament connected with dental pulp. The experimental group was allocated to three types according to the degree of lesions: mild (shadow area 10–30 mm^2^), moderate (shadow area 30–50 mm^2^), and severe (shadow area >50 mm^2^). Gingival tissues of the third molars that needed to be extracted due to impaction of five cases were collected as the control group. Sample collection: after sterilizing with 1% iodine tincture, the apical granulation tissue was scraped from the sinus tract of the affected tooth with a sterile curette under local anesthesia, and the gingival tissue of the normal control was excised. The sample was assigned to two parts: one part was quickly frozen with liquid nitrogen at −80°C for RT-PCR; another part was immediately fixed in 10% (volume fraction) neutral formaldehyde buffer solution for more than 12 hours. The samples were dehydrated by gradient alcohol, permeabilized with xylene, embedded in melted paraffin, and prepared into 4 *μ*m thick serial sections for HE staining, immunohistochemical staining, and ELISA.

### 2.3. RT-PCR

Granulation tissue of the sinus tract after chronic apical periodontitis and gingival tissue of normal control were obtained and transferred to an RNase-free 1.5 ml centrifuge tube. After adding 1 ml Trizol, the tissue was ground with a disposable grinding rod at room temperature without stirring for 5 minutes. Phenol chloroform 200 *μ*l was added, shaken, mixed, and centrifuged at 4°C and 12000 rpm × 15 minutes. The upper water sample was transferred to an additional RNase-free EP tube (approximately 500 *μ*l). An equal volume of isopropanol 500 *μ*l was added, mixed, placed at room temperature without stirring for 10 minutes, and then centrifuged at 4°C and 12000 rpm × 10 minutes. After removal of the liquid, the RNA pellet was washed with 1 ml 75% ethanol and centrifuged at 7500 rpm × 5 minutes and 4°C. After the liquid was discarded, the RNA pellet was dried in the air. RNase-free water 20 *μ*l was added to the water bath at 58°C for 10 minutes to dissolve the RNA. The sample was frozen at −70°C for further use. After isolation using Trizol reagent (Invitrogen), it was reverse transcribed into cDNA. After reverse transcription, fluorescent quantitative PCR was performed as follows: 95°C for 10 min, 94°C for 10 s, and 55°C for 30 s for 40 cycles. Starting from 60°C, the temperature was slowly raised to 95°C at 0.2°C per second, and the solubility curve was drawn. Three parallel controls were set in each group. Three experiments were performed for each sample. The relative expression was calculated by the 2^−ΔΔCt^ method.

### 2.4. ELISA

Serum sample 100 *μ*l and standard solution 100 *μ*l were incubated at 37°C for 2 h and washed four times with PBST. Diluted antibody solution 100 *μ*l was added and incubated at 37°C for 1 h, and washed four times with PBST. Diluted HRP solution 100 *μ*l was added and incubated for 40 min at 37°C, and washed four times with PBST. TMB substrate 100 *μ*l was added and incubated at 37°C in the dark for 15–20 min. Finally, 100 *μ*l of stop solution was added, and the absorbance was immediately measured at 450 nm and 630 nm using the microplate reader. The linear regression curve of the standard substance was drawn, and the concentration value of each sample was calculated in accordance with the curvilinear equation, and the content of cytokine was calculated in each tissue.

### 2.5. Immunohistochemical Staining

The sections were sequentially placed in xylene I for 8 min, xylene II for 8 min, xylene III for 8 min, anhydrous ethanol I for 5 min, anhydrous ethanol II for 5 min, 85% alcohol for 5 min, 75% alcohol for 5 min, and then washed with running water for 2 min. Heat-induced antigen retrieval was performed. After self-cooling, the slides were placed in PBS (pH 7.4) and washed three times with shaking on a decolorizing shaker, each for 5 min. A histochemical pen was employed to draw a small circle 3–4 mm apart from the tissue along the outline of the tissue, and then a sufficient amount of PBS was added. Endogenous peroxidase 50–100 *μ*l was added to each slice and incubated for 25 min at room temperature. The slides were washed three times in PBS (pH 7.4) each for 5 min. BSA 3% was added dropwise to evenly cover the tissues, and then blocked at room temperature for 30 minutes. After dropping the primary antibody on the slices, the slices were placed flat in a humid box and incubated overnight at 4°C in a refrigerator. After washing three times in PBS (pH 7.4) each for 5 min, the supersensitive rabbit mouse universal secondary antibody (HRP-labeled) was dropped to cover the tissue and incubated at room temperature for 50 min, followed by the same wash as above. Freshly prepared DAB chromogenic fluid (prepared with the ratio of dilution and concentrated solution 1000 : 50) was added. The color development time was controlled under the microscope. The positive reaction presented brownish yellow. The sections were washed with pure water to terminate the color development. Subsequently, the sections were counterstained with hematoxylin, washed with running water, dehydrated and dried with alcohol, permeabilized with xylene, and mounted with neutral resin.

### 2.6. Measurement of the Periapical Bone Resorption Area of the Experimental Group

The oral CBCT analysis software was utilized to measure the shadow of the periapical lesions. The maximum diameter was measured three times. The area was calculated by the formula, and the average was taken.

### 2.7. Statistical Analysis

SPSS 20.0 statistical software was used to analyze and process the data (*x* ± *S*). Independent sample *t*-test was applied to compare the difference in TGF-*β* expression between the normal control and experimental groups. One-way analysis of variance was used to analyze the difference among experimental samples with different degrees of inflammation. Spearman's correlation was employed to analyze the correlation between gene and protein expression and the degree of inflammation. A value of *P* < 0.05 was considered statistically significant.

## 3. Results

### 3.1. Comparison of mRNA and Protein Expression of TGF-*β* between the Two Groups

The TGF-*β* mRNA and protein expression levels in the experimental group were significantly different from those in the control group (*P* < 0.05), and the expression of both in the experimental group was higher than that of the control group, as shown in Table 1.

### 3.2. Correlation between TGF-*β* Expression and the Degree of Periapical Lesions in the Experimental Group

Spearman's correlation analysis showed that the degree of lesions was positively correlated with TGF-*β* mRNA (*r* = 0.691, *P*=0.003) but not correlated with TGF-*β* protein (*r* = 0.164, *P*=0.631), as shown in Table 2.

### 3.3. Correlation between TGF-*β* Expression and Different Lesions

There were significant differences in TGF-*β* mRNA expression between groups (*F* = 3.921, *P*=0.046, *P* < 0.05), as shown in Table 3. There was no significant difference in TGF-*β* protein expression between groups (*F* = 0.068, *P*=0.934, *P* > 0.05), as shown in Table 3. RT-PCR results showed that the expression of TGF-*β* mRNA in the experimental group was higher than that in the control group (*P* < 0.01), as shown in Table 2. As shown in Figure 1, the case group was divided into mild inflammation group (a), moderate inflammation group (b), and severe inflammation groups (c) according to the degrees of periapical lesions. The expression of TGF-*β* in the mild inflammation group (12.100 ± 1.343) was lower than that in the moderate and severe inflammation groups (16.211 ± 3.975, 17.633 ± 1.555, *P* < 0.05), as shown in Table 4. There were significant differences between the mild inflammation group and the moderate and severe inflammation groups (4.111 ± 1.751, 5.533 ± 2.243, *P*=0.035, 0.028), as shown in Table 4. TGF-*β* mRNA expression in the moderate inflammation group was lower than that in the severe inflammation group (*P* > 0.05), as shown in Table 4. The difference between the two groups was not statistically significant.

### 3.4. Results of Immunohistochemistry

The results of positive staining of TGF-*β* protein in the experimental group and the control group are shown in Figure 2. The positive staining of TGF-*β* protein presented diffuse brownish yellow in the cytoplasm. In the experimental group, a large number of TGF-*β* protein-positive cells infiltrated in the granulation tissue of the sinus tract (Figure 2(c)). Diffuse brown-yellow was visible in the cytoplasm of most macrophages and neutrophils (Figure 2(d)). In the control group, positive expression of TGF-*β* protein was occasionally seen in macrophages of the gingival tissue (Figures 2(a) and 2(b)).

## 4. Discussion

Chronic apical periodontitis, a chronic inflammation of the periapical tissue, is caused by long-term infection and pathogenic irritants in the root canal. A previous study has exhibited that bacteria, such as *Prevotella nigrescens* and *Porphyromonas spp.* in the root canal, are strongly associated with the formation of fistulas after chronic apical periodontitis [13]. The major clinicopathological manifestations of chronic apical periodontitis contain the formation of inflammatory granulation tissue and inflammatory bone resorption. When local lesions are active, fibrous components in the granulation tissue decrease, inflammatory cells and capillaries increase, and many osteoclasts are produced, causing injury to a large area of bone. Osteoclasts connected to the bone matrix by combining with integrins change and polarize the cytoskeleton structure, thereby realizing osteoclast function [14]. To remove pathogenic microorganisms and necrotic tissue in the root canal, and to promote bone tissue repair, root canal therapy is currently the major therapy in clinic. It is difficult to make an effective assessment of its efficacy in a short period, so long-term observation of the efficacy is clinically meaningful. Present studies have revealed that the five-year success rate of root canal therapy reaches 84.6% [15, 16]. Inflammatory bone resorption is an immune response regulated by various cytokines, among which interleukin-1, tumor necrosis factor alpha, and nuclear factor-*κ*B ligand receptors (RANKL) have been confirmed to only play an important role in bone resorption [17, 18]. Nevertheless, clinical prognostic indicators for the diagnosis of periapical periodontitis have not yet been concluded, which makes it impossible to judge the treatment at this stage. Therefore, this study sought to explore the relationship between TGF-*β* and the occurrence and development of chronic apical periodontitis by observing the changes of TGF-*β*.

The TGF-*β* superfamily is a family of factors with more than 30 members, mainly consisting of TGF-*β*, bone morphogenetic protein, activin, and inhibin [19]. The signaling pathways transduced by members of the TGF-*β* superfamily regulate tissue growth and development by affecting cell proliferation, differentiation, and migration [20]. Through the downstream Smad signaling pathway, TGF-*β* plays a vital role in coupling bone formation and bone resorption and maintaining normal postpartum bone homeostasis. With consecutive in-depth studies of classic Smad pathway of TGF-*β*, bone resorption could be delayed by changing the binding sites of signal molecules, by dephosphorylation, by importing other molecules, and by interfering with the binding of ligands and receptors. Some scholars have considered that TGF-*β*1 can induce CD4^+^T cells to differentiate into iTreg cells and can inhibit bone marrow mesenchymal stem cell apoptosis and tissue engineered cartilage resorption [21].

The results of RT-PCR and ELISA demonstrated that the mRNA and protein levels of TGF-*β* were significantly higher in the experimental group than those in the normal control group, suggesting that TGF-*β* may be an important factor involved in the occurrence and development of chronic apical periodontitis. We conducted a Spearman's correlation analysis to explore whether the expression of TGF-*β* mRNA and protein is correlated with the degree of disease. The results displayed that the degree of chronic apical periodontitis was positively correlated with TGF-*β* mRNA, but not with TGF-*β* protein. These findings indicated that compared with normal gingival tissue, as the degree of periapical lesions increased, TGF-*β* mRNA level increased. However, TGF-*β* protein level in the serum of the experimental group did not increase with the degree of periapical lesions. This may be due to the high sensitivity of TGF-*β* mRNA in granulation tissue, while it is affected by other factors in the serum. Because the sensitivity of plasma TGF-*β* at the protein level is very limited, TGF-*β* protein level cannot be used as an index to judge the degree of apical periodontitis. To further understand the precise relationship between TGF-*β* mRNA and the degree of lesions in the experimental group, the experimental group was divided into three levels according to the degree of lesions: mild (shadow area 10–30 mm^2^), moderate (shadow area 30–50 mm^2^), and severe (shadow area >50 mm^2^). The experimental results confirmed that in the range of mild to moderate inflammation, TGF-*β* mRNA expression tended to increase with the expansion of the lesion, but there was no statistical difference between the moderate and severe inflammation groups. This may be due to the great activation of the body's defense mechanisms in the severe inflammation stage, which tends to regenerate and repair tissues. The study concerning animal models of spontaneous inflammatory apical inflammation demonstrated that with the abnormal activation of bone osteoclasts, a large amount of TGF-*β* was released from the bone matrix, and numerous mesenchymal stem cells were recruited through the classical pathway, and osteoblast precursor cells were accumulated in the bone marrow cavity [22]. Under the action of excessive TGF-*β* signal, these precursor cells cannot successfully migrate to the bone surface for normal differentiation in order to couple with osteoclast bone resorption and eventually lead to phenotypic changes of subchondral bone, which in turn induces corresponding changes in articular cartilage [23]. Local suppression of the TGF-*β* pathway can successfully reverse the pathological changes in the alveolar bone, thereby remarkably delaying the periapical lesions, and dramatically promoting the healing of the periapical alveolar bone resorption. TGF-*β* overexpression leads to the disconnection of the alveolar bone during bone reconstruction, which results in the pathological changes in the alveolar bone and the periapical lesions of the alveolar bone. In the experiment, TGF-*β* level increased after chronic apical periodontitis, and the expansion of bone resorption proved this point.

Immunohistochemical results demonstrated that only a few cells in normal gingival tissue were positive for TGF-*β* staining. In granulation tissue of the sinus tract with chronic apical periodontitis, the number of positive cells for TGF-*β* staining increased; neutrophils, macrophages, and lymphocytes were present in positive cells. Some studies have confirmed that the expression of macrophages in periodontal inflammation increased, and the conversion from M2 phenotype to M1 phenotype may be the core step that mediates granulation tissue formation and periapical alveolar bone tissue destruction. Macrophages can produce inflammatory mediators and matrix-degrading enzymes to make the bone destruction active [24, 25]. When the bone fracture reaches a certain level, the area of the shadow around the apex can be roughly read on the X-ray film. TGF-*β* can be expressed and secreted by macrophages. A previous study pointed out that TGF-*β* in PMF disease could be derived from macrophages in the bone marrow, and antibodies targeting TGF-*β* could suppress bone marrow fibroblast proliferation and type I collagen expression, which provides a research basis for clinical targeted therapy of PMF [26].

In summary, TGF-*β* exerts crucial effects on the occurrence and development of chronic apical periodontitis, and its mechanism may involve multiple signaling pathways. This team will use TGF-*β* inhibitors to stimulate osteoclast precursor macrophages, to suppress TGF-*β* expression, to establish animal models of periapical periodontitis with TGF-*β* knockout mice and clinical patients as subjects, to verify the consistency of TGF-*β* changes in cells, animals, and humans with apical periodontitis, and to further investigate the influence and mechanism of signaling pathways on bone destruction in apical periodontitis with sinus tract. This provides new ideas and sites for the treatment of periapical periodontitis and the remodeling of alveolar bone.

## Figures and Tables

**Figure 1:** Different degrees of periapical lesions in patients with chronic apical periodontitis: (a) mild; (b) moderate; and (c) severe).

**Figure 2:** Immunohistochemical results of TGF-*β*. (a, b) Positive expression of TGF-*β* in the normal control group. (c, d) Positive expression of TGF-*β* in the experimental group (a, c × 100; b, d × 400).

**Table 1:** Comparison of TGF-*β* mRNA and protein levels between the experimental and control groups (*x* ± *s*).

Group	mRNA (*n*)	Protein (*n*)	TGF-*β* mRNA	TGF-*β* protein	*t*	*P* value
Experimental	16	11	15.193 ± 3.621^*∗*^	8512.066 ± 2204.619^*∗*^	15.087	≤0.001
Control	5	4	1.102 ± .515	6301.928 ± 1207.867	2.461	0.033

^*∗*^ *P* < 0.05, vs. control group.

**Table 2:** Correlation between TGF-*β* expression and the degree of periapical lesions in the experimental group.

TGF	*n*	*r*	*P* value
TGF-*β* mRNA	16	0.691	0.003
TGF-*β* protein	11	0.164	0.631

**Table 3:** Relationship between the expression of TGF-*β* and the degree of different lesions.

TGF	*n*	F	*P* value
TGF-*β* mRNA	16	3.921	0.046
TGF-*β* protein	11	0.068	0.934

**Table 4:** Relationship between TGF-*β* mRNA expression and different degrees of inflammation (*x* ± *s*).

Grade of inflammation	*n*	Mean	Standard deviation	*P* value
Mild	5	12.100	1.343	0.035
Moderate	8	16.211	3.975	0.028
Severe	3	17.633	1.555	0.506

## Data Availability

The data used to support the findings of this study are available from the author upon request.
